# Effect of Platelet-Rich Plasma on Bone Healing in Immediate Implants Analyzed by Cone Beam Computerized Tomography: A Randomized Controlled Trial

**DOI:** 10.1155/2021/6685991

**Published:** 2021-03-13

**Authors:** Aleshba S. Khan, Naauman Zaheer, Abdul M. Zaigham, Maliha Shahbaz, Usman Zaheer, Mohammad Khursheed Alam

**Affiliations:** ^1^Department of Prosthodontics, Islamabad Medical and Dental College, 45400, Pakistan; ^2^Department of Oral Biology, Institute of Dentistry, CMH Lahore Medical & Dental College, National University of Medical Sciences, 54810, Pakistan; ^3^Department of Prosthodontics, Institute of Dentistry, CMH Lahore Medical & Dental College, National University of Medical Sciences, 54810, Pakistan; ^4^Department of Oral Biology, Rashid Latif Medical College, 54600, Pakistan; ^5^Department of Orthodontics, Lahore Medical & Dental College, 53400, Pakistan; ^6^Preventive Dentistry Department, College of Dentistry, Jouf University, 72721, Saudi Arabia

## Abstract

The possibility of platelet-rich plasma (PRP) on the improvement of bone and adjacent tissue recovery has previously been validated. However, there is insufficient data supporting the use of platelet-rich plasma to improve the healing of bone and adjacent tissues around an implant in the oral cavity. The purpose of this randomized controlled trial was to observe the effect of platelet-rich plasma (PRP) concentrate on marginal bone loss and bone density around immediate implant placement using Cone Beam Computerized Tomography (CBCT). This clinical study was conducted over a period of six months on 12 subjects, who were equally categorized into two groups. Group I was the control, whereas the subjects in Group II received PRP therapy at the surgical site. All subjects were given a standard treatment with a single implant system (DIO UFII hybrid sandblasted acid-etched implants). Inserted implants were analyzed through CBCT, and records were registered at baseline, at the 12^th^ week before functional loading and the 26^th^ week after functional loading. The bone loss was calculated at the proximal (mesial and distal) side of the implant and bone density at baseline, 12^th^ week, and 26^th^ week after implant placement. SPSS version 23.0 was used for statistical analysis of data. The changes in bone levels were measured and compared between the two groups using the Mann–Whitney *U* test, with no significant difference. Bone density was analyzed by an independent sample *t*-test, *p* value ≤ 0.05 was considered statistically significant. Again, no significant difference in bone density was observed between both groups at all three instances. Therefore, it can be concluded that local injection of PRP after immediate implant placement did not show any decrease in marginal bone loss or improvement in bone density. This trial is registered with NCT04650763.

## 1. Introduction

Tooth loss is a distressing experience and affects the quality of life [1]. Implants provide a fixed replacement option improving the patient's confidence and have psychological benefits [1, 2]. Bone requires approximately 2 to 3 months for remodeling after extraction of the tooth, and it has been suggested healing time of common commercial titanium implants is 3-6 months before loading becomes clinically feasible [1, 3]. The elaborate treatment planning, followed up with the surgical procedure as well as the use of a removable prosthesis temporarily till definitive prosthetic replacement, decreases the willingness of the patients who tend to prefer early restoration of function and esthetics [1].

The immediate implant placement in an extraction socket seems to have some benefit when compared to delayed implant placement, such as less time and reduced surgical procedures [2, 4]. Previously, many studies have concluded that immediate implant placement minimizes bone resorption by maintaining the periodontal architecture [2, 5, 6]. However, recent clinical studies have reported increased failure rates due to a decrease in primary stability and a reduction in bone volume around immediately placed implants, suggesting that it did not effectively prevent vertical and horizontal changes in ridge volume [2, 7, 8]. Nonetheless, there was no significant difference in bone loss between the two groups [8].

The prognosis of immediate implants may be compromised by the presence of residual dental infection or any bony defect. However, at sites with intact socket walls of the alveolar bone intact have been reported to have a similar survival rates to that of implants placed into healed ridges [2, 8].

Platelet-rich plasma (PRP) is an autologous concentrate of platelets in a minute amount of plasma [9]. It is considered a first-generation concentrate using calcium glutamate/thrombin to activate coagulation and an anticoagulant solution of citrate phosphate dextrose adenine (CPDA) [10, 11]. After activation by thrombin or calcium chloride, the platelets in PRP release various essential growth factors documented to be produced by platelets [12]. These growth factors consist of 3 isomers of platelet-derived growth factors (PDGF*αα*, PDGF*ββ*, and PDGF*αβ*), 2 transforming growth factors-*β* (TGF*β*1 and TGF*β*2), epithelial growth factor, and vascular endothelial growth factor [2, 9]. Once used locally, platelet concentrates increase the production of osteoprogenitor cells, initiate osteoblast activity, accelerate epithelialization of the gingiva, promote cell recruitment at the site of surgery, and stimulate angiogenesis [9]. Apart from these benefits, PRP may play anti-inflammatory and analgesic roles during the early period after surgery, as documented in some randomized clinical studies [13, 14]. The inclusion of leukocytes in PRP releases VEGF and TGF that, again, improves chemotaxis and angiogenesis [10], mainly due to the control of the inflammatory process by anti-inflammatory cytokines IL-4, IL-6, and IL-10 also having an antimicrobial potential [10]. Antimicrobial activities of platelet concentrates against some oral microbes reduce the incidence of postoperative infection, which is an advantage when treating cases with an infected postextraction sockets [14].

However, there is no consensus on whether or not platelets must be previously activated before their application and with which agonist [12]. Thrombin and calcium chloride, which are aggregation inducers, are used to activate platelets and stimulate degranulation, causing the release of the growth factors. Some authors activate platelets, whereas others apply platelets without previously activating them, arguing that better results are obtained [12]. While working on this trial, there was still no definitive outcome as to the adverse effects of using thrombin to release growth factors. Recent studies found that such aggregators are not necessary because at the time of administration the platelets are automatically released and ready to exert their function [12]. Thus, thrombin was replaced with normal saline for this study [2, 12]. Moreover, this technique/protocol of preparing and using PRP is generally followed in Pakistan's hospitals for clinical uses. So, PRP was the preferred choice for this study.

PRP containing platelet growth factors has been used widely in multiple procedures, and evidence showed improved tissue healing, but its positive effect on hard tissue healing still needs more research [15, 16]. Some clinical studies reported controversial results in the bone formation and marginal bone preservation around immediate implants when platelet-rich plasma was used [2, 9]. Thus, further research is needed to determine the influence of PRP on the bone.

The objective was to study the effect of platelet-rich plasma concentrate on marginal bone loss and bone density in immediate implant placement through CBCT in a human clinical trial.

## 2. Methodology

A randomized control trial was conducted at the Department of Prosthodontics, Institute of Dentistry, CMH, Lahore Medical College, over a period of six months from October 2018 till March 2019. Approval was taken from the ethical committee of the Institute of Dentistry, CMH, Lahore Medical College (Reference #466/ERC/CMH/LMC), and the study was registered in ClinicalTrials.gov (NCT04650763). Twelve systemically healthy subjects above the age of twenty were selected including both genders. The sample size was estimated by using 95% confidence level, 80% power with an expected mean change in bone loss for PRP and control group in 12-week time as 0.27 ± 0.07 and 0.65 ± 0.28, respectively [1]. Subjects included were patients maintaining good oral hygiene, having adequate bone quantity at the implant site, and patients requiring extraction and replacement of at least one tooth by a prosthesis supported on the implant with or without the application of PRP.

Patients with active infection around the implant site, immunocompromised state, with current major systemic disease (uncontrolled diabetes, rheumatoid arthritis, etc.) or oral pathologies, history of bleeding disorders or on anticoagulant therapy, or patients on bisphosphonates were excluded from the study. Subjects who were physically and mentally challenged (lack of manual dexterity) and those who were noncompliant for regular visits and follow-ups were also excluded from the study. Personal information of the patients was kept confidential. Informed consent was obtained for documentation and public presentation of their clinical data.

All chosen individuals who agreed to be part of the research received standard treatment with a single implant system (DIO UFII implants, hybrid, sandblasted and acid-etched surface). Randomization of subjects was done (6 in each group) by nonprobability consecutive sampling. Another researcher allocated random numbers to the participants for the purpose of concealment and to avoid bias. Half of the participants were assigned odd numbers, and half were assigned even numbers randomly. Odd numbers were added in Group I, the control group (non-PRP group), and even numbers were added in Group II (PRP group), which was a test group that received PRP therapy. There were 6 cases in each group. Analyses of inserted implants were done as per CBCT. Clinical records were noted at baseline and at each follow-up visit after 12 weeks before functional loading and 26^th^-week follow-up after functional loading.

The data was measured for bone loss at the mesial and distal sites and bone density at baseline, 12-week, and 26-week time. The changes between baseline and 12 weeks, baseline to 26 weeks, and 12–26 weeks were measured and compared between the two groups (Figure 1). The data was significantly deviating from normality for bone loss at both sites for at least one of the groups. Mann–Whitney *U* test was applied to compare two groups. The data for bone density was normal, so an independent sample *t*-test was applied. *p* value ≤ 0.05 was considered significant. SPSS version 23.0 was used for statistical analysis of data.

## 3. Procedure

### 3.1. Preparation of PRP

The PRP was made ready for use just before placement at the surgical site. 9 ml of blood was taken from the antecubital vein and put in the test tube containing 3.8% trisodium citrate acting as an anticoagulant [2]. An automated blood cell centrifuge was utilised to extract PRP. The product code ORG having premarket review showing Center for Biologics Evaluation and Research (CBER). The submission type is 510(k) with regulation number 864.9245. The device is class 2 with total product life cycle (TPLC) code report. The sample of blood was immediately centrifuged at 5800 rpm for 8 minutes at room temperature to separate poor platelet plasma from RBCs and PRP and then centrifuged at 2400 rpm for an additional 5 min to obtain further separation of PRP from RBCs [2]. After centrifugation, the top buffy coat was collected into a syringe and injected or mixed with saline to form a liquid solution, to inject at the surgical site [2, 12].

### 3.2. Surgical and Prosthetic Phase

During surgery, a full thickness mucoperiosteal flap was reflected [17], and the osteotomy was done through sequential drilling for both groups. To determine the size of the implants, presurgical radiographic evaluation and diameter apical to crestal bone along with length of socket was analyzed through CBCT [18, 19]. The implant was inserted in the osteotomy site until the crest module of the fixture was at the same level with the crest of the margin. The immediately prepared liquid solution of PRP was injected on the labial aspect between the implant surface and buccal alveolar wall [2]. Then, sutures were placed to close the flap. PRP has osteoconductive properties which imply that cell growth and differentiation factors from the surrounding bone must be recruited and directed toward the surgical site to accomplish their regenerative action. Osteoinductive mediators serve as crucial elements necessary to achieve a proper osseointegration, as they stimulate various stages of bone regeneration [2].

After 12 weeks, CBCT was taken before functional loading. Soft tissue thickness and interocclusal space were evaluated with WHO periodontal probe for placement of an appropriate size of the abutment on the fixture. A torque of 30 N cm was used for the placement of the abutment after a one-stage nonfunctional immediate prosthetic protocol. Instructions on the maintenance of hygiene and soft diet plan were emphasized. Three months after insertion of the implant, the definitive prosthesis was cemented with zinc phosphate cement, and the excess cement was wiped immediately after crown placement and further removed with an explorer after setting.

### 3.3. Radiographic Evaluation

The crestal bone changes were measured at the time of implant placement (baseline), before functional loading, at the 12^th^ week, and the 26^th^ week after functional loading. CBCT (Planmeca Romexis 5.1.0.4) with voxel size 200 *μ*m was used for analysis and measurement.

Marginal bone loss was measured in millimetres from the reference line, the maximum height of the crest module to the first visible bone level to implant contact on the mesial and distal sides [20]. Two perpendicular lines were dropped from the reference line on the mesial and distal aspect of the implants to the first bone-to-implant contact. Bone loss was compared in the individual patients in a sagittal view as mesial and distal sides through CBCT at the 12^th^ and 26^th^ weeks (Figure 2).

The baseline reference direction for the short and long axes was set at the bottom of the inner basic lamellae of the cortical bone at the coronal portion of the implant and the implant surface. To assess the bone density at the coronal portion of the implants, three-dimensional bone morphometrical analyses were done on a region within 1 mm from the baseline of the long axis in the apical direction and within 0.6 mm from the baseline of the short axis. The short axis will further be divided into two regions: from the surface to 0.2 mm (near zone) and from 0.2 to 0.6 mm (far zone). Bone density was evaluated in an axial view of CBCT in grey value by Hounsfield unit [21] (Figure 3).

## 4. Results

The average bone loss at mesial site was 0.37 ± 0.80 in the control group between baseline and 12^th^ week, while in the PRP group it was 0.03 ± 0.08. The comparison between the two groups was insignificant, with a *p* value of 0.461. The largest change at the mesial site was observed in the control group in 26-week time from baseline, while the bone loss in the PRP group for the same duration was 0.07 ± 0.10 still, the difference was statistically insignificant with a *p* value of 0.212. At the distal site, the mean bone loss was 0.07 ± 0.016 between baseline and 26^th^ week while it was 0.0 between 12 and 26 weeks in the PRP group, which was insignificant compared to the control group with *p* values 0.290 and 0.140, respectively. There was no significant difference in changes in bone density between the two groups with *p* values > 0.05 for all three instances (Table 1).

## 5. Discussion

The bone quality and quantity around implants affect the osseointegration phase and influence soft tissue architecture [1]. Assessment of marginal bone levels and bone density as well as soft tissue has become a basic element of the evaluation of the implant patient and is usually a significant tool for the assessment of implant success [1, 20, 21].

The amount and quantity of bone around the implant can be enhanced by providing a stimulus to improve the regenerative potential of the tissue [1, 2]. Multiple growth factors are expressed during tissue healing tissue. Therefore, the introduction of growth factors through platelet concentrate can act as healing agents to accelerate both peri-implant soft and hard tissue repair [2].

The present study did not show any significant difference in marginal bone loss and bone density, following PRP's use with immediate implant placement, compared to the control group. Other studies have also concluded that no difference was found in PRP and non-PRP groups on hard tissue assessment [2] and that the effect of PRP on the height of bone was not significant [22, 23]. Despite the nonsignificant outcomes, when we look closely at the graphical data, along with radiographic parameters though CBCT radiographs, PRP did show promising effects in reducing marginal bone loss and improving bone density which implies that PRP therapy does improve osseointegration [15] and bone density around the implant surface, thus leading to better stability [24]. Other studies also reported significant results when PRP was used and concluded that it enhances osseointegration and reduces marginal bone loss [25, 26].

Nevertheless, statistical analysis showed nonsignificant results which might be because of small sample size and because PRP was injected primarily on the labial aspect between the implant surface and buccal alveolar wall, rather than moistening the implant surface with PRP before placement of implant in the socket, as done by other researchers [15, 24]. Other reasons for the differences in results might be because the preparation systems are not the same [27]; the centrifuge machines vary in revolutions per minute [27], challenges in obtaining a homogenous composition of PRP as there is variation between different people [28] and it is not noticeably clear how will this affect the stem cell behavior in different individuals [29].

## 6. Conclusion

Based on the radiographic images of CBCT and the graphical data obtained from this study, PRP's effects on marginal bone loss and bone density around immediate dental implants were promising. Although the results were statistically insignificant, the increased sample size might improve the validity of the results and achieve statistically significant results in the future. In further studies, bone density can be analyzed through a Dual Energy X-ray Absorptiometry (DEXA) scan of the mandible after the use of PRP on the implant surface or in the extraction socket before implant placement to better understand the effects of PRP on the bone. More research can be done to gather long-term and robust evidence on PRP's success so that it can be incorporated in regular practice after implant placement to improve the prognosis of treatment.

## Figures and Tables

**Figure 1:** Bone loss and bone density at mesial and distal sites in two groups at baseline, 12 weeks, and 26 weeks.

**Figure 2:** Marginal bone loss: (a) day 0, baseline control group; (b) 12 weeks, control group; (c) 26 weeks, control group; (d) day 0, PRP group; (e) 12 weeks, PRP group, (f) 26 weeks, PRP group.

**Figure 3:** Bone density: (a) day 0, baseline control group; (b) 12 weeks, control group; (c) 26 weeks, control group; (d) day 0, PRP group; (e) 12 weeks, PRP group; (f) 26 weeks, PRP group.

**Table 1:** Comparison of bone loss at mesial and distal sites and bone mineral density between the two groups at different times.

Variable	Change between	Group				*p* value
		Control		PRP		
		Mean	SD	Mean	SD	
Measurement of bone loss at mesial site	Baseline–12 wk	0.37	0.80	0.03	0.08	0.461^a^
	Baseline–26 wk	0.43	0.77	0.07	0.10	0.212^a^
	12–26 wk	0.07	0.10	0.03	0.08	0.523^a^
Bone loss at distal site	Baseline–12 wk	0.07	0.10	0.07	0.16	0.673^a^
	Baseline–26 wk	0.17	0.20	0.07	0.16	0.290^a^
	12–26 wk	0.10	0.17	0.00	0.00	0.140^a^
Bone mineral density	Baseline–12 wk	69.25	65.46	28.37	83.74	0.368^b^
	Baseline–26 wk	378.27	270.86	233.10	212.08	0.326^b^
	12–26 wk	309.02	234.53	204.73	159.30	0.389^b^

^a^The *p* value is calculated by Mann–Whitney *U* test. ^b^The *p* value is calculated by independent sample *t*-test. SD: standard deviation.

## Data Availability

The pictures of data used to support the findings of this study are included within the article. The entered Excel sheet data of this study are available from the corresponding author upon request.

## Supplementary Materials

Supplementary 1 Supplementary file 1: CONSORT 2010 checklist.

Supplementary 2 Supplementary file 2: CONSORT 2010 flow diagram.
